# Securitization Concept and Its Application to Environmental Problems in the Kurdistan Region: Prospects and Obstacles

This article has been retracted.

**DOI:** 10.1155/2022/8122568

**Published:** 2022-05-26

**Authors:** Salam Abdulqadir Abdulrahman, Nusret Sinan Evcan

**Affiliations:** Cyprus International University, Nicosia, Cyprus

## Abstract

Environmental pollution has caused a wide range of problems across the globe. Various studies have focused on worldwide water and environmental issues and their effects on human health and political and social aspects. This article, on the other hand, discusses soil, water, and air pollution as well as the overuse of water resources. This study then discusses these problems as a security issue in the Kurdistan Region of Iraq (KRI) context. This research adopts a qualitative approach. It reviews the results of previous studies on soil, water, and air pollution in KRI to demonstrate the causes and scale of the problem. It then explores securitization by looking at the main components of the concept and how they can be applied and what needs to be adjusted. Results of the study have shown that pollution is widespread, water is overexploited, and there is a lack of an effective response by the Kurdistan Regional Government (KRG). In addition, in the KRI context, securitization is state-centered, meaning that the country's decision-makers play an important role in securitizing issues. The Kurdistan Regional Government, that is, the securitizing actor, should do more on the speech act, and this should be preceded by substantial political, economic, and psychological changes. Finally, the government must also enforce strict water control to support its water policies.

## 1. Introduction

The overthrow of Saddam Hussein in 2003 was the beginning of a new era in Iraq. It came after years of war, economic sanctions, and international isolation. Iraq was then able to do trade with the outside world and make deals with foreign companies. This opportunity was quickly seized in KRI. Having been outside the administrative authority of the Iraqi government since 1992, KRI was better organized to take advantage of the new opportunity. KRI increased its volume of trade, mainly importing goods and services from other countries, especially from Turkey and Iran, and expanded investment in the construction and energy sectors. Its economy started to grow, together with the expansion of its urban centers. Many people from rural areas migrated to the cities, and numerous people got jobs in the public sector or registered with KRG to receive a monthly allowance. These changes were spurred on by the rise in income for the KRG, which was mostly from oil exports.

Yet these changes have had serious consequences for the environment. Increasing waste matters and wastewater from the expanding urban centers pollute soil and render both the surface water and groundwater unsuitable for drinking and even irrigation, and there is an increasing need for land to be used as landfills and dumpsites. In KRI, waste and wastewater are largely not recycled or treated. The soil is also polluted by the growing oil industry and other industrial activities. Water is polluted by human activities, and water as a resource is overexploited. The demand for water from expanding urban areas and agriculture is rising to an unprecedented level. This has led to the overwithdrawal of both groundwater and surface water. And the air quality in KRI is rapidly deteriorating. An unprecedented number of cars on the roads, together with a huge number of privately owned electricity generators and other industrial activities, have turned the air quality in KRI into one of the worst in the world.

The damage to the environment continues apace, but no significant recovery program is in place. As we demonstrate, immediate and exceptional measures should be taken by the government that can be achieved by transforming the existing regime of practice and allocating sufficient human and financial resources for as long as and as much as it takes, i.e., to securitize the matter and elevate it to the top of the government agenda. This is securitization in action, and it can be done in KRI if certain things happen, like the political organization of society, the economic system, and the psychological state of people, to make the securitization work.

This paper is divided into three sections. In the first section, we study the pollution of soil, water, and air in KRI and focus on its causes. We also study the overexploitation of the natural resources of water. In the second section, we look at the securitization concept and explain its components. The researchers also clarify how it can be applied to the situation. In the third and final section, the researchers look at the political, economic, and psychological impediments to active securitization. The researchers end the paper by talking about how one of the most important problems in KRI is not getting enough attention but is still very important and highlight the main problems that still need more advanced solutions in this matter.

The Kurdistan Region of Iraq is situated in the northeast of Iraq. It consists of four governorates: Erbil, with an estimated population of 2.2 million; Sulaymaniyah, with an estimated population of 2.1 million; Duhok, with an estimated population of 1.6 million; and Halabja, with an estimated population of 115.4 thousand. Since 1992, KRI has been a selfadministered area in Iraq. Its legal status is recognized in the new Iraqi constitution, which was approved in a national referendum in 2005, two years after the overthrow of the former Iraqi dictator. It covers an area of about 40 000 km^2^. The Kurds constitute the majority of its population, along with other ethnic and religious minorities. KRI's neighbors are Iran on the east, Turkey on the north, and Iraq on the west and south [1, 2]. KRI is the only place in the world where the Kurds have a degree of autonomy. The Kurds are the largest nation in the world without a state. Following the fall of the Ottoman Empire in the early 20th century, their land was split up between Turkey, Iran, Iraq, and Syria.

The aim of the research is to highlight serious environmental problems in KRI, namely, the pollution of the main environmental components, the pollution of soil, water, and air, and the overexploitation of water resources, and explain how they have happened. It is also to argue for the relevancy of securitization to the problem, but also how securitization as a concept and process will need to be attuned to the situation.

## 2. Problem, Methodology, and Contribution

To state the problem of the research, we can say that the overthrow of Saddam Hussein's regime in Iraq in 2003 was the beginning of a new era in the country; the decade-long economic and trade sanctions were lifted so Iraq could once again interact with the outside world for trade and other transactions. This opportunity was best seized by the semiautonomous KRI. KRI had been selfadministrated since 1992, which meant that it had functioning government institutions prior to the regime change.

The new situation allowed trade with the outside world and the acceleration of economic growth, which also meant the growth of urban areas. However, these developments have caused significant damage to the KRI environment. The KRG has largely ignored the effects of economic and urban development on the environment, especially the pollution of soil, water, and air and the damage to the water resources.

The scale of the damage is huge and should not be ignored anymore, and it requires rapid action and effective solutions to be taken by the authorities. This research paper looks at the problem and assesses it from a securitization perspective, meaning that the government's priority must change to the environment and the country's financial and human resources must be diverted to solving the urgent environmental threats, the pollution of the main environmental components, and the overexploitation of water. The research also looks at the main obstacles to securitization and argues that when applied to local environmental problems, the nature of the securitization process will change and so the concept needs to be reassessed.

This research adopts a qualitative approach. It reviews the results of previous studies on soil, water, and air pollution in KRI to demonstrate the causes and scale of the problem. It then explores securitization by looking at the main components of the concept and how they can be applied and what needs to be adjusted.

The research will have two main contributions. The first contribution comes from its attempt to use securitization in specific areas of the environment, namely, pollution and resource overexploitation. And the second contribution comes from the adjustments that need to happen to the process of securitization when applied to local environmental problems and the implications of this for the concept.

### 2.1. Environmental Problems in KRI

In this section, we highlight two main areas of environmental problems in KRI: first, the pollution of the soil, water, and air; and second, the overexploitation of water resources. Both problems are getting worse by the day, and they threaten the well-being of people and the sustainability of the environment. Threats like these constitute security issues [3] since they are directly related to the survival or well-being of the people. Therefore, they require to be treated urgently and with the utmost effort.

Soil pollution in KRI has three main sources. The first source is industrial activities in general and the oil industry in particular [4]. Heavy metals (i.e., arsenic, copper, chromium, cadmium, cobalt, iron, manganese, molybdenum, nickel, lead, and zinc) have been found in large quantities in the soil around industrial areas as well as in urban centers [5], and extraction, refining, and transportation of oil have created immense pollution [6]. There are many oil refineries, licensed and unlicensed, in KRI that occupy vast areas of land and discharge their effluents into the environment. These activities cause soil contamination and destroy agricultural lands on a large scale [7]. Another source of soil pollution is the transport of crude oil and petroleum derivatives by tanker trucks to and from neighboring countries. There are around 5,000 oil tanker trucks on KRI roads every day, and accidents often happen because of bad roads, faulty trucks, or bad driving [8]. Some of these accidents result in the spillage of huge volumes of oil and the contamination of wide areas of land.

The second source of soil pollution is municipal solid waste, mainly in urban areas [9]. Urbanization and a change in lifestyle for many people have led to an increase in the consumption of all sorts of goods and, consequently, an increase in waste material. Almost all the solid waste ends up in open dumpsites or landfills [10], and some of these places are not very far from the residential areas. In some dumping lands, the solid wastes are burned haphazardly, with the air pollution distribution of a rotten odor [11]. There are also unauthorized dumpsites in many areas. More and more land is being used for increasing municipal solid waste.

The third source of soil pollution is waste from urban centers and other residential areas. Untreated wastewater (there is no system in place to separate wastewater into grey and black, it is all mixed) mixes with the rivers or creeks and continues traveling through the land. Wastewater released by sewerage pipes or tunnels is a source of surface and subsurface soil pollution in KRI. The wastewater of Sulaymaniyah city, which pours into the Tanjaro River, is an example in that regard [12]. Other areas that do not have sewerage systems, including all the villages, rely on cesspits for the disposal of their waste. The cesspits allow the wastewater to spread through and pollute the soil as well as the groundwater.

The water is increasingly polluted in KRI. The sources of surface water pollution are wastewater and industrial discharges, including discharges from oil refineries and agricultural farmlands. Untreated wastewater from these sources mixes with rivers and lakes [13]. The Dukan Reservoir, the largest lake in KRI and the main source of drinking water for Sulaymaniyah governorate, including Sulaymaniyah city, is contaminated with heavy metals to an alarming level [14]. Heavy metals are nonbiodegradable and cause various serious diseases when accumulated in living tissues [15]. The quality of Sulaymaniyah's water has been declining over the past years, and it is expected to decline further owing to the insufficient preventive measures by the local authorities [16]. The Tanjaro River, Qlyasan Stream, and Darbandikhan Reservoir in Sulaymaniyah governorate are some other examples for contamination of surface water with heavy metals. Tanjaro and Qlyasan receive untreated domestic and industrial waste before they join the Darbandikhan Reservoir, which is the second largest lake in KRI and the source of drinking water for hundreds of thousands of people. Abdul Hameed M. et al. [17], Salih Majid et al. [18, 19], and Ahmed Khwakaram [20] say that the water in the reservoir is not safe for people to drink.

The drinking water of the Duhok governorate is another example. It is contaminated and not suitable for drinking. It includes the city of Duhok, the largest urban center in the governorate and the third-largest city in KRI. The city's drinking water comes from the Duhok Dam, which is polluted by socioeconomic activities including agriculture. The water receives some treatment before it is pumped to consumers, but it is still polluted with fecal bacteria [21–23]. It is then sent into the Duhok Valley without any treatment, where it is used for irrigation of fruits and vegetables and to water animals before it reaches the Mosul Dam after a 24-kilometer journey [24]. It is then sent into the Mosul Dam after that.

Groundwater is another main source of both drinking water and irrigation. It is the only source of water in many areas of KRI. This resource can become polluted by agricultural, urban, and industrial wastes that leak into underlying aquifers [25]. KRI groundwater is polluted in some areas by these sources. Sulaymaniyah groundwater, its well-water and karez-water (subterranean water), for example, is not potable because of leakage from sewage and other contaminants. The situation is worse for groundwater in those places that are adjacent to polluted rivers, streams, or sewage outlets [26]. Many places near oil refineries have very dirty groundwater [27].

Another example of groundwater pollution is the groundwater of the Makhmur plain, which is the largest cropland area in the Erbil governorate and has a sizable population. According to one study [28], the water is not safe for people to drink.

Air is being increasingly polluted in KRI, with many health consequences for people [29]. Highly toxic gases and toxic metal elements are being released into the air from industrial activities in general and oil activities in particular (Meena B.I. and Omar K.A. [30]). Toxic gases with heavy metals in the air are also attributed to heavy traffic density in the urban centers and on the roads [5]. Heavy traffic density has also been linked to soil pollution in urban areas [31]. KRI has no tram, train, or underground train. It has a bus service, but it is suited to malls and operates only in limited areas and often without a timetable. Many people rely on their own cars for transportation.

Almost all the existing vehicles in KRI run on gasoline or diesel. This contributes to increasing air pollution. Lead emissions from cars have a high level of lead, a heavy metal. Tetraethyllead is added to gasoline in KRI “to improve its quality and to increase its octane number,” but with huge consequences for human health and the environment [32].

Another main source of air pollution is private electricity generators operating in residential neighborhoods. In KRI, consumers generally receive electricity from two sources: national and private. National electricity means the electricity that comes from the state-owned power plants, and private electricity means the electricity that is supplied by privately-owned electricity generators operating in the residential areas. Each generator supplies power to some hundred houses or shops. In KRI, national power is not constant; it often cuts out, especially on cold and hot days when demand for electricity is high. Private generators fill the gap. They supply power, sometimes up to 12 hours a day, and, as a result, release huge amounts of CO2, NOx, SO2, CO, solid particulates, and CB into the air [33]. Therefore, the generators constitute a major source of air pollution, which, combined with the gases emitted by cars, oil tanker trucks, and factories, often creates a layer of black clouds over the cities [34]. People in positions of power can be made to see the seriousness of the problem and be persuaded to get the public to agree with them [35].

Another serious environmental problem is the overexploitation and overconsumption of natural resources, mainly water. The surface water, which comes from precipitation and international rivers, is not properly harvested. Only a small amount is kept in few lakes, and a lot of it is wasted when it is sent to homes or farms [36, 37].

Groundwater is being seriously overexploited and degraded in KRI. Groundwater is heavily used for drinking and irrigation in most areas in KRI. Digging tools and drilling machines have made it easy for many people to get the tube or artesian wells on their farms or even in their back yards. It is easy to obtain a government license for digging a well, but if it is not obtained, people still dig wells because they know that they can easily get away with it; generally, there are no legal consequences. Moreover, the government is also responsible for degrading the groundwater. It considers that groundwater can easily be accessed to satisfy short-term needs. Consequently, tens of thousands of water wells have been constructed all over the KRI. The excessive withdrawal of their water has markedly lowered the groundwater table. For example, the groundwater in the Erbil province has fallen by half from 2000 to 2015 [38]. This shows that withdrawal has been much higher than recovery and that water has been used in an unsustainable manner [39].

Unsustainable usage of water resources is a serious environmental problem in KRI. There are also some other factors that contribute to the deterioration of water, namely, the climate change factor and controlling the flow of the transboundary rivers by upstream Iran and Turkey. These factors add to the water shortage in KRI. The water security in KRI is at great risk [40–42].

All in all, the environmental problems in KRI are getting worse, and there are no plans by KRG to meet the scale of the problem [43]. In the following section, we study the securitization concept, which has existed since the end of the Cold War. It is held to be useful for tackling nonconventional threats, whether socioeconomic or environmental. We explain the concept and look at its different parts, and we say that the concept needs to be changed to serve a specific purpose in a specific area, like KRI's environmental problems.

### 2.2. Securitization of Environmental Problems

Securitization can mean different things in different fields. In the legal sector, for example, it means a “transaction or scheme, whereby the credit risk associated with an exposure or pool of exposures is tranche (divided into parts)” [44]. Securitization is the process of turning an issue into a security issue, putting it in the security realm or on the security agenda so that it can be dealt with in a different way [45, 46].

Security was considered to be a matter of international relations. It was understood to be about interstate rivalries; for example, a state perceives an existential threat, usually of a military type, arising beyond its borders; therefore, it has to repel it by all the means at hand [47]. This is the realist approach to security. It is now considered to be a narrow understanding of what constitutes a security issue or what constitutes national security. Securitization of the environment takes a broader view of security than usual, and it is best pursued at the state level. Environmental securitization at the international level does not stand a chance. It boomeranged in the case of the UK's and Netherlands' attempts to securitize climate change [48–50].

Environmental issues were among the nontraditional (socioeconomic) issues to be transformed into the security realm in the second half of the twentieth century [51, 52]. Problems in this sector could no longer be ignored, such as the “loss of biodiversity and habitat degradation of water and soil” [53]. Environmental issues slowly and increasingly gained ground in the second half of the twentieth century as a matter directly related to the sustainability of modern life [54, 55]. In 1987, the United Nations General Assembly called this type of security “environmental security.” According to Ruth Noorduyn and Wouter T. de Groot [56], civil society groups began to focus on environmental issues, and this led to a general, revolutionary change in Europe in the late 20th century.

Environmental problems refer to the changes in the Earth's atmosphere, soil, and water, such as air, water, and soil pollution and the degradation of their quality and quantity; excessive use of natural resources; and the consequences of those changes for people and the ecosystem. The KRI presents many such problems. Securitization in this context means framing environmental problems as threats and successfully transforming them into the security agenda, which will in turn “become the hegemonic discourse type in government policy” and call for “policies of exception,” according to Olaf Corry [57]. This means that some threats are highlighted over others and that the intellectual and material resources at the disposal of the state will be employed to deal with them [58, 59].

Securitization as a process has four main components: the securitizing actor, the referent subject, the referent object, and the audience. The securitizing actor is the top decision-maker in the country who has an acceptable degree of legitimacy (i.e., discursive legitimacy as there are no universal values for legitimacy) and that person might be supported or convinced by the functional actors or support actors such as NGOs to securitize a threat. The actor makes a convenient speech, called a speech act, which has to be understood in the broader social environment and believed to be effective in dealing with the issue at hand, i.e., with the referent subject, which is portrayed as a threat to the referent object by using security-laden words to convince the audience to accept the new approach. The referent object must also have a legitimate and genuine claim to survival. This can be anything important to the audience, or it can be the audience themselves, as in the case of environmental problems. It is important that the audience must be convinced that the action the securitizing actor intends to take is necessary to deal with the threat [55, 58–60].

The audience's conviction gives legitimacy to the securitizing actor to go ahead with the proposed action. In the words of Balzac, the greater the audience's persuasion, the greater the ability of the leaders to carry out the securitization process [47]. The conviction element may imply that securitization can truly happen only in democratic systems where the legitimacy of the political leaders comes from the public's consent. This might indicate that securitization is not applicable in nondemocratic political systems where political leaders rule with force and do not need the audience's consent [61]. But this is not very accurate. Leaders of the nondemocratic and totalitarian political systems still seek their people's consent in different ways [62].

In the context of KRI, the securitizing actors are the country's decision-makers; above them is the Prime Minister, who holds the highest office in the land; and the functional actors are the civil society groups, prominent individuals, and the media, which have a significant influence on the country's decision-makers as well as the audience. The referent subjects are the environmental problems we have studied in the previous section. The referent objects are the people who live in KRI, especially those who are most affected by the environmental problems and the environment itself. Considering the environment as a referent object is necessary because the insecurity of an entity will jeopardize the survival of another entity and, consequently, the survival of all. The audience is the people and the country's legislators. The latter is more formal in its support of the securitization move, while the former is more informal in its support. Last but not least, it will require a lot of state resources to deal with the growing environmental problems [47, 52, 53, 59, 63–65].

Here, we need to state that the proposed securitizing actors in KRI are responsible for creating the very threat that they now have to guard against and that the audience is also responsible for creating the threat that they need to be protected from. The referent objects include both the audience and the securitizing actors who need to be protected from the threat. The environment, which is considered to be the source of the threat, is in fact an object to be protected from the threat; it is a victim too [66].

The environmental problems in KRI are material and objective, and they directly affect people. These factors help to make a stronger argument for their securitization [49, 59, 67]. Some experts say that in order for a securitization process to work, there must be real-world factors like material evidence that can be used to make people aware of the size of the threat and how important it is to act quickly.

When securitization is completed and the problems have been dealt with successfully, there can be a reverse process by which the securitized matter would be returned to normal politics, where it will be treated in a manner similar to the treatment of other problems [68]. Because the government cannot spend all of its resources on one thing, like the environment, for very long, this is a step that must be taken. Other things need to be looked at, and the state must be ready to deal with any new problems that come up, so this is a good thing to do.

### 2.3. Obstacles to Securitization

Environmental securitization in KRI is not only a matter of clarifying and applying the concept theoretically. There are certain obstacles on the ground that hamper the success of the process: the political organization of society and events around the KRI borders as political obstacles, the patron-client economy as an economic obstacle, and the recent history of KRI as a psychological obstacle. Securitization cannot happen successfully as long as these obstacles are present.

The KRI's political organization or political system is created and maintained by two ruling political armed parties. They are the Kurdistan Democratic Party (KDP) and the Patriotic Union of Kurdistan (PUK). Since the end of their civil war in 1998, the KDP has controlled the northern and western parts of Erbil governorate and all of Dohuk governorate, while the PUK has controlled the southern and eastern parts of Erbil governorate and all of Sulaymaniyah and Halabja governorates. The two parties share power in one government, the KRG, but at the same time, they continuously build up more military and intelligence power and control revenue sources for each party in their zone of control. KDP has an upper hand over government affairs because the government cabinet is based in Erbil City, which is in KDP's zone of control. The two parties maintain sizable military, security, and intelligence agencies, and they own dozens of media outlets. The two parties, directly and indirectly, support different political and social groups in return for their loyalty. For KDP and PUK, what matters most of the time is their own power and survival, and they are prepared to do anything in that regard. This means that issues like environmental problems do not matter much to them [50, 69, 70].

The political system of KRI is one of the leading reasons for the neglect of environmental problems. It allows a large portion of the country's revenues to go to the ruling political parties. Members of the ruling parties who occupy high governmental posts are preoccupied with personal gains and their parties' security and survival, and they are less interested in issues that concern the nation as a whole. This has led to a situation where KRG does not get sufficient income to manage its own administrative affairs.

The second political obstacle is events around the KRI borders. KRI is located in a region characterized by intense military security and armed rivalries and conflicts. All of the KRI's neighbors, Iran, Turkey, Syria, and Iraq, are concerned about their security and are engaged in military confrontations with their adversaries near the KRI's borders [71, 72]. Syria fights many rebel groups [73] and Iraq fights remnants of ISIS [74]. This state of affairs has a considerable impact on the decision-making in KRI regarding what problems constitute security threats and what issues should be given the highest attention. In the wider region, there is a lot of support for military security, which makes it less likely that nonmilitary issues will be resolved.

The economic impediment to environmental security is the result of political organization. Over the past three decades, the ruling parties have used the country's resources to buy people's loyalty. The policy they pursued was that both the parties, each in their zone, recruited many people in the public sector while there were no real vacancies for many of them. They also registered many people to receive monthly allowances from the government. Hundreds of thousands of people went on the KRG payroll. Many become “ghost employees,” meaning employees without a job or a post but still paid. Besides, some employees receive more than one salary from the government as they are registered with different names or with the same name but in different government departments, and some of those people receive a salary from the government and a salary from the ruling political parties. Furthermore, the ruling parties have salaries or allowances for their own members. Businesses, small and big, are also dependent on the support of the ruling parties [70, 75–77].

In total, more than a million people out of the 6 million people living in KRI are recipients of monthly salaries, pensions, or allowances [78]. This situation is very costly for the government to maintain; sometimes all the national revenues collected in a month are not enough to fully pay all those who are on the government payroll in that month [79]. This is at a time when KRG has a real problem with collecting the national revenues completely because of the division of KRI into two zones of control. Accordingly, with regard to the securitization of the environment, things look bad: there might not be enough financial resources at the government's disposal for environmental problems. Another thing to keep in mind is that the people who get money from the government are not likely to agree to any securitization move that could affect their monthly payments.

The third obstacle to environmental securitization in KRI is psychological. It is the result of many wars and conflicts in the area. The Kurdish liberation movement from the 1940s and the continuing struggle and armed conflicts with the successive Iraqi regimes have turned KRI into a battleground. Besides, the eight-year Iran-Iraq war created further destruction and caused many deaths. The chemical attack on the town of Halabja and the Anfal campaign genocide, which together killed more than 180,000 Kurdish civilians, are two more examples of war and conflict in KRI [9, 80, 81]. People, specifically the elderly generation, are familiar with the sound of gunshots and artillery shelling, and images of war and violence are lodged in their memories. These events, together with the ongoing military conflicts around the KRI borders, have made military threats constant and far and away from the most recognizable kind of threat. The environment is displaced by the attacks on its human residents.

## 3. Conclusion

Soil, water, and air pollution and water overexploitation in KRI create existential threats to people. This research has argued that these problems need to be solved in an effective and urgent manner. KRI's environmental problems have been growing for quite a long time. They constitute real threats to the lives and wellbeing of people and also to the ecosystem. The solution can best be achieved when these problems are transformed into the realm of security, where life-threatening issues receive the highest attention from the government, i.e., when they are securitized.

Securitization is security in motion. It is security in broad terms to include threats from unconventional sources alongside the military. The military capability of the enemy is no longer counted as the only source of threat to the inhabitants of a country. There are many other threats that are no less dangerous to life or the quality of life than military threats, such as poverty, hunger, deadly diseases, denial of one's ethnic or religious identity, or one's language, culture, tradition, or way of life. These threats are existential in the sense that they threaten the very existence of life or the dignity of the targeted population. Soil, water, and air are the main components of the environment, and when they get bad, they make life less good and it is hard to keep up in the long run.

KRI's environmental problems need an urgent and effective solution. We proposed securitization as a mechanism for that solution and clarified who should do it and how. We proposed that the securitizing actor be the country's top decision-makers, most importantly the Prime Minister of KRG; the functional actors, those who initiate and/or support the securitization act, to be the civil society groups, media outlets, and prominent individuals; the environmental problems to be designated as the referent subject; and the referent object to be the people living in KRI who should be freed from the problems. The people are also the audience who, through their representatives in the parliament but also the media and other outlets, give their consent or rejection to a proposed securitization act [82]. We rationalized that the securitizing actors are at the same time referent objects in the sense that they are affected by environmental problems. We say that the people who now need to be protected are themselves a threat to the environment. This is because most modern environmental problems are caused by people being careless with the environment and misusing its resources.

Environmental securitization carries the promise of solving the KRI environmental problems in an urgent and effective manner. The process can begin now and the roles can be distributed as we have proposed above, but it will not be successful unless several main obstacles on the ground are removed: political, economic, and psychological. In other words, these obstacles need to be treated first. The political obstacle is related to the political organization of KRI and also to the security situation in the border areas. The political organization allows the ruling parties, KDP and PUK, to pursue narrow party interests, prolong the division of KRI into two zones, and use the national revenues for their own benefits. This means that power struggles, party security, and interests take precedence, while other issues are pushed to the sidelines. The economic obstacle is the result of the KRI clientele economy, whereby the national revenues largely go to the ruling parties and the government employees and allowance receivers. This means that fewer financial resources are available for environmental securitization. Lastly, the situation near the KRI borders and the people's memory of war and conflict affect the way people classify threats.

For the securitization of environmental problems to happen in KRI, the speech act, which is considered the first step, must be preceded by significant political, economic, and psychological improvements; the improvement of the political and economic systems; and efforts to be made to minimize the effects of war on people's minds. This is mainly the task of the securitizing and functional actors. Securitization is, of necessity, a long and unpredictable process [83–88].

## Data Availability

Data are available upon request.
